The article "Variable Heights Influence Lower Extremity Biomechanics and Reactive Strength Index during Drop Jump: An Experimental Study of Male High Jumpers" was published in 2021. Journal: J Healthc Eng.

# Variable Heights Influence Lower Extremity Biomechanics and Reactive Strength Index during Drop Jump: An Experimental Study of Male High Jumpers

**DOI:** 10.1155/2021/5185758

**Published:** 2021-11-30

**Authors:** Zehao Tong, Feng Zhai, Hang Xu, Wenjia Chen, Jiesheng Cui

**Affiliations:** ^1^College of Physical Education, China University of Mining and Technology, Xuzhou, Jiangsu, China; ^2^Department of Medical Imaging, Xuzhou Medical University, Xuzhou, Jiangsu, China; ^3^National University of Singapore 119077, Singapore

## Abstract

**Introduction:**

This study finds the lower limbs' reactive strength index and biomechanical parameters on variable heights.

**Objective:**

This research aims to reveal the effects of drop height on lower limbs' reactive strength index and biomechanical parameters.

**Methods:**

Two AMTI force platforms and Vicon motion capture system were used to collect kinematic and dynamic signals of the lower limbs.

**Results:**

The drop height had significant effects on peak vertical ground reaction force and peak vertical ground reaction force in the extension phase, lower limbs' support moment, eccentric power of the hip joint, eccentric power of the knee joint, eccentric power of the ankle joint, and concentric power of the hip joint. The drop height had no significant effects on the reactive strength index. Reactive strength index (RSI) had no significant correlations with the personal best of high jumpers. The optimal loading height for the maximum reactive strength index was 0.45 m.

**Conclusion:**

The optimal loading height for the reactive strength index can be used for explosive power training and lower extremity injury prevention.

## 1. Introduction

Drop jump (DJ) is always a core part of plyometric training for high jumpers. It has also been used to find the effect of variable heights on lower limbs' biomechanical parameters and reactive strength index (RSI). Kipp et al. found the effect of variable heights on the biomechanical indicator and RSI in male basketball players, but RSI, vertical stiffness, and other parameters were unaffected by drop height [1]. Wu et al. indicated that DJ height marked impacted the peak of vertical ground reaction force (vGRF) in male paratroopers [2]. Peng found that negative power and vGRF at higher loading heights were higher than low heights in college students [3]. It is known that the same DJ height has different effects on the RSI and biomechanical parameters of various subjects, so it is necessary to determine an appropriate loading height of DJ for each sport event.

Current research studies reported that DJ height for the maximum RSI could enhance sport performance. Ramirez-Campillo et al. reported that optimal loading height for the RSI could significantly increase the 20 m sprint of soccer players by 7 weeks of intervention, but did not point out the DJ height for the RSI [4]. Boullosa et al. selected the optimal loading height for the RSI during warm-up, which improved the CMJ performance of long-distance runners, but failed to increase 1000 m performance [5]. Smirniotou et al. found that the RSI was highly correlated with sprint speed in young sprinters, but did not apply the result to intervention [6]. Hennessy and Kilty revealed that BDJ index has a significant correlation with 30 m and 100 m performance in female athletes, but did not use for further training [7]. It is quite clear that optimal loading height for the RSI is hard to improve the personal best (PB) directly for most of sports, but it should be stressed that the ideal PB is related to sport performance.

The article "Variable Heights Influence Lower Extremity Biomechanics and Reactive Strength Index during Drop Jump: An Experimental Study of Male High Jumpers" was published in 2021. Journal: J Healthc Eng.

High jump includes fast run-up takeoff and high flight height. Studies showed that RSI can effectively evaluate the ground contact time and flight height. Flanagan et al. [8] and Ebben and Petushek reported that RSI has high reliability on the evaluation of lower limbs' explosive power [9]. Markwick et al. found that RSI can effectively assess the plyometric training of male basketball players [10]. Meanwhile, Louder et al. confirmed the high internal validity of the RSI [11]. Some research studies believed that PB was affected by vertical height of high jump. Mateos-Padorno et al. reported that vertical displacement in the sagittal plane has a high correlation with PB [12]. Viitasalo and Aura found that the vertical height of the jumpers was increased at the game season [13]. Therefore, the improvement of RSI may be helpful for PB. In addition, high jumpers were always tortured by lower extremity injury. Schmitt et al. believed that most of elite high jumpers have injured ankle and knee joints in the takeoff leg [14]. Schmitt et al. reported that a certain proportion of high jumpers suffered by hip arthrosis [15]. Schmitt et al. found that the jumpers with ankle injury have a low radiological score [16]. It should be emphasized that inappropriate training results in injury [17].

To our knowledge, no studies found the effects of variable heights for high jumpers. Many studies showed that RSI could significantly improve the sprint and CMJ performance, but did not clarify the correlations between the RSI and the PB of high jumpers. Therefore, the aim of this study was to investigate the effects of variable drop heights on vGRF, RSI, joint power, and moment of lower limbs, find the correlations between RSI and PB, and determine the optimal loading height for the maximum RSI. Hypotheses include the following: (1) drop height had significant effects on the reactive strength index and biomechanical parameters. (2) The correlation between the RSI and PB would be significant.

The article "Variable Heights Influence Lower Extremity Biomechanics and Reactive Strength Index during Drop Jump: An Experimental Study of Male High Jumpers" was published in 2021. Journal: J Healthc Eng.

## 2. Methods

Ten high jumpers were recruited (males: age: 20.7 ± 2.32 y, training background: 5.1 ± 1.51 y, weight: 72.33 ± 5.36 kg, height: 1.89 ± 0.04 m, and personal best: 2.065 ± 0.04 m). Vicon motion capture system (Vicon, UK) and AMTI HPS400600 force platforms (AMTI, USA) were used to collect kinematic and dynamic signals of the lower limbs. Plyo Soft Box was used for the DJ test (Escape Fitness, UK). The warm-up protocol included 10 min of jogging at a moderate self-selected pace [5] and 5 min of static stretching for each leg. After hearing the “start” order, raise the dominant leg, naturally lean forward, and drop freely. When the feet touch the ground, the subject must jump vertically as fast as possible. Requirements of effective DJ were as follows: do not move center of gravity upwards after leaving the box. Both feet should touch the ground at the same time. Jump upwards with full strength, and keep both hands on hips [18]. Vicon motion capture system was used to capture kinematic signals of the lower limbs at a frequency of 100 Hz. According to the pasting scheme of Plug-In Gait Lower-Limb Ai 2.3 Marker [19], 28 reflective markers were pasted on the bony landmarks of the lower limbs. 24 markers were reserved for motion capture. The location and name of the markers are shown in Figure 1.

Vicon Nexus (v.2.10.1, Vicon, UK) was used to synchronously collect kinematic and dynamic data. Vicon Nexus was also used to identify the reflective markers during static calibration and export them in a C3D format. Visual 3D (v.6.01.36, C-Motion, USA) was used to build bony models of human lower limbs and process original dynamic and kinematic signals to obtain dynamic and kinematic data of lower limb joints. The marker trajectory and analog data were filtered with a fourth-order low-pass Butterworth filter at 6 Hz and 15 Hz, respectively, to reduce the noise in the signals [20]. Reactive strength index (RSI) was worked out as the ratio of flight height and ground contact time. The processed data were calculated using the following formula [21, 22]:

(1) $$\begin{array}{c} Hf=\frac{1}{2}g{\left(\frac{Tf}{2}\right)}^{2}\left(m\right),\\ \text{RSI}=\frac{Hf}{Tc}. \end{array}$$

The average value for three effective DJs at the same height was calculated. By quadratic polynomial regression analysis, the effects of drop height on the biomechanics parameters and RSI of the lower limbs were obtained. One-way repeated measure analysis of variance (ANOVA) was used for comparison of differences and selected the significant variables of them for Bonferroni correction. The maximum average value was taken from each group as the optimal loading height for the RSI. By Pearson's test, the correlations of RSI and PB were investigated. The above data were processed with SPSS (v. 25.0, IBM, USA).

The article "Variable Heights Influence Lower Extremity Biomechanics and Reactive Strength Index during Drop Jump: An Experimental Study of Male High Jumpers" was published in 2021. Journal: J Healthc Eng.

## 3. Results

Table 1 shows the result of quadratic polynomial regression analysis. The drop height significantly affected vGRF (*P* < 0.001) and vGRFep (*P* < 0.001), lower limbs' support moment (*P* < 0.05), eccentric power of the hip joint (*P* < 0.05), eccentric power of the knee joint (*P* < 0.001), eccentric power of the ankle joint (*P* < 0.001), and concentric power of the hip joint (*P* < 0.001). It has no significant effects on the hip extension moment (*P* > 0.05), knee extension moment (*P* > 0.05), ankle plantarflexion moment (*P* > 0.05), and RSI (*P* > 0.05).  Table 2 shows the result of one-way repeated measure analysis. vGRF (*P* < 0.001), vGRFep (*P* < 0.001), hip extension moment (*P* < 0.05), knee extension moment (*P* < 0.05), eccentric power of the hip (*P* < 0.05), knee (*P* < 0.05), and ankle joint (*P* < 0.05), and concentric power of the hip joint (*P* < 0.05) have statistical significance at 0.3 m, 0.45 m, 0.6 m, and 0.75 m.

Table 3 reflects mean values (±SD) and the result of Bonferroni correction during DJs. Relative to the drop height of 0.3 m, vGRF (*P* < 0.008) increased significantly at 0.45 m, 0.6 m, and 0.75 m. vGRF at the DJ height of 0.75 m was significantly larger than at 0.45 m and 0.6 m (*P* < 0.008). Compared with the drop height of 0.3 m, vGRFep (*P* < 0.008) increased significantly at 0.6 m and 0.75 m. Relative to the DJ height at 0.3 m, the hip extension moment (*P* < 0.008) increased significantly at 0.6 m. The eccentric power of the hip joint (*P* < 0.008) at 0.75 m was significantly larger than at 0.3 m, 0.45 m, and 0.6 m. Compared with DJ height at 0.3 m, eccentric power of the knee joint (*P* < 0.008) was increased significantly at 0.45 m, 0.6 m, and 0.75 m, while it increased significantly at 0.6 m relative to 0.3 m and 0.45 m (*P* < 0.008). The eccentric power of the knee joint (*P* < 0.008) at the DJ height of 0.45 m was significantly larger than at 0.3 m. Relative to the drop height of 0.3 m, eccentric power of the ankle joint (*P* < 0.008) increased significantly at 0.6 m and 0.75 m, while it increased significantly at 0.75 m relative to 0.45 m (*P* < 0.008). The eccentric power of the ankle joint at 0.6 m was significantly larger than at 0.3 m (*P* < 0.008). Compared with the drop height of 0.3 m and 0.45 m, the concentric power of the hip joint (*P* < 0.008) increased significantly at 0.75 m, while it increased significantly at 0.6 m relative to the drop height of 0.3 m (*P* < 0.008). The RSI (0.17 ± 0.04) was the largest average in the group, so the optimal loading height for the RSI was 0.45 m. The result of Pearson's test reflected that RSI has no significant correlations with PB (*r* = 0.149, *P* > 0.05).

The article "Variable Heights Influence Lower Extremity Biomechanics and Reactive Strength Index during Drop Jump: An Experimental Study of Male High Jumpers" was published in 2021. Journal: J Healthc Eng.

## 4. Discussion

vGRF and eccentric joint power were significantly affected by drop height in the lower limbs. Studies have found that vGRF was affected by drop height, which was further demonstrated in this research [2, 3, 23, 24]. According to the law of free-fall, the higher drop height converted gravitational potential energy into kinetic energy, and a greater momentum was generated at the landing phase, so a greater vGRF can be generated at a higher drop height. Eccentric joint power was increased with the increase of DJ heights; it is caused by the neuromuscular adaptation [25]. It means that high jumpers can keep the shorter contact time at the landing phase. Therefore, the eccentric joint power of high jumpers was increased with DJ height.

Drop height had a significant impact on vGRFep, low limb support moment, and concentric power of the hip joint. vGRFep represented the level of active muscle contraction [26]. The jumpers could achieve maximum vGRFep at a lower DJ height, caused by short-term stretch-shortening cycle (SSC). It means more active muscle contraction can be generated in shorter coupling time during this process. In addition to the short-term SSC, short-latency reflex (SLR) also cannot be ignored in the active contraction of the lower limbs. Taube et al. found that drop jump controlled SLR and stretch reflex activation of the lower limb [27]. Komi and Gollhofer reported that when the drop height was controlled within 0.2 m–0.6 m, the SLR of the soleus was positively correlated with the drop height and significantly decreased at 0.8 m [28]. It indicated that the muscle-tendon complex was increasing stiffness and storing more elastic energy by the increasing SLR and stretch reflex level at a suitable range of DJ heights. When the loading height exceeds the appropriate value, stretch reflex and SLR activation were decreased, resulting in the low stiffness of the muscle-tendon complex for reducing the excessive impact [29]. Active contraction was limited by the low SLR and stretch reflex activation, presenting a decrease in vGRFep at excessive drop heights. Meanwhile, the concentric power of the hip joint was increased with DJ height, which may be related to the technical requirements of high jump because the jumpers performed takeoff several times when extending the hip during their training. Avela et al. believed that high jumpers could adapt the high impact during DJ [25]. Kim suggested an elite jumper to improve the extension strength [30]. Therefore, high jumpers could quickly extend the hip and generate the greater concentric power of the hip joint when performing DJs under excessive heights.

The article "Variable Heights Influence Lower Extremity Biomechanics and Reactive Strength Index during Drop Jump: An Experimental Study of Male High Jumpers" was published in 2021. Journal: J Healthc Eng.

The result indicated that lower limbs' support moment was significantly affected by drop height and had no significant effects on knee extension moment and ankle plantarflexion moment. It was related to the neuromuscular adaptation of high jumpers to high impact loads. It indicated that high jumpers can still keep the extension of lower limb joints, even at high DJ height. Avela et al. showed that high jumpers have no significant changes in soleus H-reflex and SLR sensitivity during DJ [25]. Evidence shows that the modulation of spinal nerves could maintain the H-reflex and SLR sensitivity of the soleus at a low level under rapid stretching and high impact load and prevent the muscle-tendon complex from excessive stress in the landing phase [25, 29]. Nevertheless, joint extension of the lower limbs will result in the increase of the Achilles tendon in the landing phase. Laurent et al. found that the stiffness of the Achilles tendon in the knee extension group increased significantly at 0.2 m, 0.4 m, and 0.6 m [31]. Previous research studies showed that most of lower extremity injuries were induced by excessive stiffness. Brazier et al. reported that much lower or higher stiffness in the lower limbs leads to an increased risk of injury [32]. Choi and Cho showed that excessive joint stiffness is one of the reasons of stress fractures [33]. Faria et al. believed that excessive stiffness of the muscle-tendon is a risk factor for lower extremity injuries [34]. Therefore, high jumpers should control stiffness, when it is at an excessive level. It is important to use maximum RSI to reduce the worse effect of this special landing style (lower limbs' extension and fast takeoff) of high jumpers.

The drop height had no significant effects on the RSI, mainly due to the neuromuscular adaptation. The modulation of the muscle H-reflex and SLR sensitivity of high jumpers by upper spinal nerves showed no significant changes before and after DJ [25], while shorter landing time could be maintained at a higher drop height. The special landing strategy of high jumpers was induced by neuromuscular adaptation in the landing phase. Studies have shown that, with this special landing strategy, greater RSI and shorter contact time could be produced at the landing phase. Guy-Cherry et al. found that vGRF of the knee extension group was maximum by investigating 5 DJs at 0.4 m, and its RSI was significantly higher than that of the knee flexion group [35]. Marchetti et al. showed that the landing time of the BDJ at 40 cm was shorter than the 90° knee flexion and 135° knee flexion [36]. Struzik et al. suggested that the RSI of the BDJ group was higher than that of the CDJ group at 30 cm, 45 cm, and 60 cm [37]. Abdelsattar et al. confirmed that Achilles tendon's stiffness and ground contact time were negatively correlated; it indicated that a stiff Achilles tendon tends to result in a faster takeoff [38]. As RSI is a parameter which can evaluate the ground contact time [8] and high stiffness of the Achilles tendon decreases the ground contact time, the special landing strategy can keep the RSI when the loading height was increased. The optimal loading height for the RSI was 0.45 m, which was nearly consistent with the data of Struzik et al. [37]. It is different from Byrne et al. [39], which may be affected by gender [40], strength [41], etc.

The article "Variable Heights Influence Lower Extremity Biomechanics and Reactive Strength Index during Drop Jump: An Experimental Study of Male High Jumpers" was published in 2021. Journal: J Healthc Eng.

## 5. Conclusion

This research found the effect of drop height on some of the biomechanical parameters in the lower limbs. One hypothesis that the drop height had significant effects on biomechanical parameters was partially supported. The result of this study indicated that the drop height had significant effects on vGRF, vGRFep, lower limbs' support moment, eccentric joint power, and concentric power of the hip joint. The drop height had no significant effects on the RSI. RSI had no significant correlations with the PB of high jumpers. The optimal loading height for the maximum RSI was 0.45 m. The optimal loading height can be used for explosive power training and injury prevention.

## Figures and Tables

**Figure 1:** The location of reflective markers. (a) Location on the lower limbs. (b) Specific location of each marker.

**Table 1:** Quadratic polynomial regression analysis for variables during DJs.

S. no.	Variables	*R*	*R* ^2^	Adjusted *R*^2^	*F*	*β*	*t*	*P*	Constant
1	vGRF	0.686	0.471	0.457	33.852	8.149	7.233	**≤0.001**	27.742
2	vGRFep	0.54	0.292	0.273	15.667	−7.275	−3.958	**≤0.001**	63.006
3	Hip extension moment	0.114	0.013	−0.013	0.5	0.09	0.707	0.484	1.43
4	Knee extension moment	0.281	0.079	0.055	3.26	0.158	1.806	0.079	3.106
5	Ankle plantarflexion moment	0.171	0.029	0.004	1.141	0.111	1.068	0.292	3.035
6	Lower limbs' support moment	0.35	0.123	0.1	5.314	0.359	2.305	**0.027**	7.571
7	Eccentric power of the hip joint	0.49	0.24	0.22	12	−9.883	−3.464	**0.001**	−4.342
8	Eccentric power of the knee joint	0.676	0.457	0.443	31.985	−6.142	−5.656	**≤0.001**	−8.729
9	Eccentric power of the ankle joint	0.531	0.282	0.263	14.946	−3.563	−3.866	**≤0.001**	−4.465
10	Concentric power of the hip joint	0.589	0.347	0.33	20.171	3.556	4.491	**≤0.001**	4.519
11	Concentric power of the knee joint	0.119	0.014	−0.012	0.547	0.457	0.739	0.464	19.267
12	Concentric power of the ankle joint	0.046	0.002	−0.024	0.081	0.202	0.284	0.778	22.514
13	RSI	0.064	0.004	−0.022	0.155	0.002	0.393	0.696	0.156

vGRF: the peak of vertical ground reaction force; vGRFep: the peak of vertical ground reaction force in the extension phase; RSI: reactive strength index. *P* < 0.05 indicates significant effects, and bold is used to indicate it, which means drop height significantly affects the indicator.

The article "Variable Heights Influence Lower Extremity Biomechanics and Reactive Strength Index during Drop Jump: An Experimental Study of Male High Jumpers" was published in 2021. Journal: J Healthc Eng.

**Table 2:** One-way repeated measure analysis of variance for variables during DJs.

S. no.	Variables	Mauchly's sphericity test	*F*	*P*	Partial eta [2]
1	vGRF	0.004	47.709	**≤0.001**	0.841
2	vGRFep	0.403	27.577	**≤0.001**	0.754
3	Hip extension moment	0.043	8.059	**0.019**	0.472
4	Knee extension moment	0.005	3.752	**0.023**	0.294
5	Ankle plantarflexion moment	0.028	0.84	0.484	0.085
6	Lower limbs' support moment	0.036	2.533	0.119	0.22
7	Eccentric power of the hip joint	0.006	32.686	**≤0.001**	0.784
8	Eccentric power of the knee joint	0.01	42.591	**≤0.001**	0.826
9	Eccentric power of the ankle joint	0.482	22.819	**0.001**	0.907
10	Concentric power of the hip joint	0.174	12.905	**0.001**	0.589
11	Concentric power of the knee joint	0.057	1.179	0.336	0.116
12	Concentric power of the ankle joint	0.091	0.48	0.699	0.051
13	RSI	0.196	0.585	0.63	0.061

vGRF: the peak of vertical ground reaction force; vGRFep: the peak of vertical ground reaction force in the extension phase; RSI: reactive strength index. *P* < 0.05 indicates a significant difference, and bold is used to indicate it. The value of this index at the drop height of 0.3m, 0.45m, 0.6m, 0.75m is significantly different from each other.

**Table 3:** Mean values (±SD) with the Bonferroni correction of variables for DJs.

S. no.	Variables	Drop height			
		0.3 m	0.45 m	0.6 m	0.75 m
1	vGRF (N/kg)	35.32 ± 8.97	44.84 ± 9.53	52.31 ± 10.1*∗*#	59.99 ± 11.82*∗*+^
2	vGRFep (N/kg)	57.01 ± 13.15^#	47.7 ± 14.94	38.87 ± 10.32	35.7 ± 14.09*∗*
3	Hip extension moment (Nm/kg)	1.52 ± 0.68^	1.66 ± 0.98	1.6 ± 0.86*∗*	1.84 ± 1.1
4	Knee extension moment (Nm/kg)	3.17 ± 0.52	3.49 ± 0.53	3.74 ± 0.64	3.61 ± 0.77
5	Ankle plantarflexion moment (Nm/kg)	3.09 ± 0.61	3.34 ± 1.08	3.35 ± 0.46	3.46 ± 0.73
6	Lower limbs' support moment (Nm/kg)	7.78 ± 0.69	8.49 ± 1.32	8.69 ± 1	8.91 ± 1.36
7	Eccentric power of the hip joint (Nm/s)	−16.55 ± 11.41#	−21.92 ± 12.65#	−31.39 ± 20.8#	−46.34 ± 31.15*∗*+^
8	Eccentric power of the knee joint (Nm/s)	−15.47 ± 5.28+^#	−20.09 ± 6.43*∗*#	−27.2 ± 8.19*∗*#	−33.57 ± 10.56*∗*+^
9	Eccentric power of the ankle joint (Nm/s)	−7.93 ± 4.72^#	−11.28 ± 7.62#	−16.07 ± 6.24*∗*	−18.21 ± 7.66*∗*+
10	Concentric power of the hip joint (Nm/s)	9.2 ± 4.33	10.38 ± 4.43#	14.33 ± 5.51*∗*#	19.73 ± 7.65*∗*+
11	Concentric power of the knee joint (Nm/s)	18.9 ± 2.3	21.33 ± 3.31#	20.8 ± 5.72	20.6 ± 5.4+
12	Concentric power of the ankle joint (Nm/s)	21.99 ± 4.54	24.02 ± 7.07	23.1 ± 3.1	22.97 ± 4.93
13	RSI (m/s)	0.15 ± 0.03	0.17 ± 0.04	0.16 ± 0.03	0.16 ± 0.04

vGRF: the peak of vertical ground reaction force; vGRFep: the peak of vertical ground reaction force in the extension phase; RSI: reactive strength index. *∗*indicates a significant difference relative to 0.3 m (*P* < 0.008), + indicates a significant difference relative to 0.45 m (*P* < 0.008), ^ indicates a significant difference relative to 0.6 m (*P* < 0.008), and # indicates a significant difference relative to 0.75 m (*P* < 0.008).

The article "Variable Heights Influence Lower Extremity Biomechanics and Reactive Strength Index during Drop Jump: An Experimental Study of Male High Jumpers" was published in 2021. Journal: J Healthc Eng.

## Data Availability

Data sharing is not applicable to this article as no datasets were generated or analyzed during the current study.
